# StartReact Effects Support Different Pathophysiological Mechanisms Underlying Freezing of Gait and Postural Instability in Parkinson’s Disease

**DOI:** 10.1371/journal.pone.0122064

**Published:** 2015-03-24

**Authors:** Jorik Nonnekes, Digna de Kam, Lars B. Oude Nijhuis, Karin van Geel, Bastiaan R. Bloem, Alexander Geurts, Vivian Weerdesteyn

**Affiliations:** 1 Radboud University Medical Centre, Donders Institute for Brain, Cognition and Behaviour, Department of Rehabilitation, Nijmegen, The Netherlands; 2 Radboud University Medical Centre, Donders Institute for Brain, Cognition and Behaviour, Department of Neurology, Nijmegen, The Netherlands; 3 Sint Maartenskliniek Research, Development & Education, Nijmegen, The Netherlands; Hokkaido University, JAPAN

## Abstract

**Introduction:**

The pathophysiology underlying postural instability in Parkinson’s disease is poorly understood. The frequent co-existence with freezing of gait raises the possibility of shared pathophysiology. There is evidence that dysfunction of brainstem structures contribute to freezing of gait. Here, we evaluated whether dysfunction of these structures contributes to postural instability as well. Brainstem function was assessed by studying the StartReact effect (acceleration of latencies by a startling acoustic stimulus (SAS)).

**Methods:**

We included 25 patients, divided in two different ways: 1) those with postural instability (HY = 3, n = 11) versus those without (HY<3, n = 14); and 2) those with freezing (n = 11) versus those without freezing (n = 14). We also tested 15 matched healthy controls. We tested postural responses by translating a balance platform in the forward direction, resulting in backward balance perturbations. In 25% of trials, the start of the balance perturbation was accompanied by a SAS.

**Results:**

The amplitude of automatic postural responses and length of the first balance correcting step were smaller in patients with postural instability compared to patients without postural instability, but did not differ between freezers and non-freezers. In contrast, the StartReact effect was intact in patients with postural instability but was attenuated in freezers.

**Discussion:**

We suggest that the mechanisms underlying freezing of gait and postural instability in Parkinson’s disease are at least partly different. Underscaling of automatic postural responses and balance-correcting steps both contribute to postural instability. The attenuated StartReact effect was seen only in freezers and likely reflects inadequate representation of motor programs at upper brainstem level.

## Introduction

Postural instability is a disabling feature of Parkinson’s disease (PD), in which the underlying pathophysiology is still poorly understood. The frequent co-existence with freezing of gait (FOG) raises the possibility of a shared pathophysiology [1, 2]. There is emerging evidence that dysfunction of upper brainstem structures, in particular the pedunculopontine nucleus (PPN) and pontomedullary reticular formation (pmRF), could play a role in causing FOG [3–5]. As automatic postural responses likely arise from the pmRF [6], dysfunction of upper brainstem structures may also underlie postural instability.

Evidence for a pivotal role of dysfunctional upper brainstem circuits in patients with FOG has been provided by studies evaluating the StartReact effect. StartReact refers to the acceleration of movement onset latencies when a startling auditory stimulus (SAS) is given at the same time as the imperative ‘go’ signal in a reaction time task. Although the exact mechanism underlying StartReact and the neural structures involved are a matter of ongoing debate [7, 8], several recent studies have provided accumulating evidence for the SAS directly releasing a subcortically stored motor program, presumably from upper brainstem structures [7, 9–13]. The StartReact effect was absent in patients with severe FOG and postural instability when performing an elbow flexion movement, but was restored after PPN stimulation [3]. In a recent study we further confirmed that the StartReact effect is attenuated in freezers, but -more importantly- in a task that is known to provoke FOG (i.e. gait initiation, [5]). Postural responses to backward balance perturbations can be modified by a StartReact paradigm [14], suggesting that they are preprogrammed and potentially subject to the same triggered release which has been shown to be deficient in freezers [3]. However, SAS-induced acceleration of postural responses has not been evaluated in PD patients. Moreover, neither Thevathasan *et al*. nor Nonnekes *et al*. evaluated whether defective StartReact effects are also related to postural instability. Therefore, it remains unknown whether dysfunction of the same brainstem reticular structures may underlie both FOG and postural instability.

In the present study, we aimed to address this question by evaluating the effect of a SAS on the onset and scaling of postural responses to backward balance perturbations. As a control, we also evaluated SAS-induced movement accelerations in a simple reaction time task involving ankle dorsiflexion. We carefully selected and balanced a group of PD patients, and specifically contrasted the results between patients with evident postural instability (as identified by a positive pull test) versus those without, and between those with FOG versus those without. If dysfunction of the same brainstem reticular structures contributes to both FOG and postural instability, we should expect to see a disturbed StartReact effect in freezers as well as in patients with postural instability.

## Materials and Methods

### Participants

The present paper concerns the same participants as in our previous paper [5], except for one PD patient for whom the examination of balance responses was too burdensome. The PD group consisted of twenty-five patients, 11 with evident postural instability (Hoehn and Yahr stage 3) and 14 without evident postural instability (Hoehn and Yahr stage 2 or 2.5). Six of the patients with postural instability had freezing of gait, and this was also true for 5 of the patients without postural instability (see below for definitions). Patients were diagnosed according to the UK Brain Bank criteria [15]. Exclusion criteria were any other neurological or orthopedic disorder affecting balance, severe cognitive impairments or use of medication negatively affecting balance. Patients were measured in an OFF state, when they experienced an end-of-dose effect prior to intake of their next medication. Clinical assessment also took place in the OFF state. In addition, 15 healthy controls of similar age were included. The study was approved by the local medical ethics committee (CMO regio Arnhem/Nijmegen) and was conducted in accordance with the Declaration of Helsinki. All subjects gave their written informed consent prior to the experiment.

### Clinical assessment

PD patients were clinically assessed with the motor subsection (Part III) of the MDS-Unified Parkinson’s Disease Rating Scale (UPDRS, score/132)[16]. Postural instability was determined by the pull-test performed by JN. The pull-test was performed as described in the MDS-UPDRS [16], which is regarded as the gold standard to evaluate postural instability in PD [17, 18]. A mild pull was applied first, which was not rated and served as a demonstration. Thereafter, a quick and forceful pull was applied, which was rated. Patients with Hoehn and Yahr stage 3 were unable to recover independently, and would have fallen if not caught by the examiner. Patients with Hoehn and Yahr stage<3 were able to recover unaided. Patients also completed the New Freezing of Gait Questionnaire (N-FOGQ, score/33)[19]. Additionally, they performed a series of walking tests to objectively verify subjects as freezers or non-freezers [20, 21]. These tests included eight rapid axial 360° turns in both directions and walking with 25% of the preferred step length (at a normal pace, and as rapidly as possible). Based on the detailed physical examination, 11 persons were classified as ‘freezers’, and the 14 other patients were classified as ‘non-freezers’ as they did not show FOG-episodes during examination, and never experienced subjective gluing in daily life (except for one patient with sporadic gluing in daily life, but who never manifested FOG during repeated and detailed neurological examinations). The N-FOGQ revealed that all freezers had more frequent and more severe FOG during the OFF-medication state. Lastly, global executive function was assessed with the Frontal Assessment Battery (FAB, score/18).

### Experimental setup and protocol

#### Postural responses

Participants stood on a moveable platform that could suddenly translate in the forward direction, resulting in a backward balance perturbation; we will refer to the direction of the balance perturbation [22]. Participants stood with their arms alongside the trunk. Platform movements comprised an acceleration phase (300 ms), a constant velocity phase (500 ms), and a deceleration phase (300 ms). We used perturbations with an acceleration of 1.5 m/s^2^. This intensity required all participants taking one or more steps to prevent falling. Participants were instructed to respond to the balance perturbations as they would do in daily life. Participants underwent 16 backward balance perturbations and consecutive trials were at least 20 seconds apart. In 25% of the balance perturbations a startling auditory stimulus (SAS) was given through binaural earphones at the start of the translation of the platform. The SAS (50 ms white noise, 116 dB sound pressure level linear fast (measured with Investigator 2260 and Artificial Ear B&K 6cc type 4152, Bruel and Kjaer, Nærum, Denmark)) was generated by a custom-made noise generator and was randomized over the trials. Subjects wore a safety harness that was attached to the ceiling and prevented them from falling.

#### Simple reaction time task

This task served to verify whether the pattern of results in the postural perturbations would also apply to a different type of movement. The results of the freezers versus non-freezer comparison have been reported in our previous paper [5], but here we will also compare patients with and without postural instability. The task involved subjects performing a simple reactive ankle dorsiflexion movement. Participants sat in a chair that was positioned 2.5 meters in front of two arrays of light-emitting diodes (LEDs; 11x8 cm, 3 cm apart). Illumination of the first LED array served as a warning signal and participants were instructed to initiate ankle dorsiflexion as soon as the second LED array was lit (‘go’ signal). Patients performed the task with their most affected side and healthy controls with their right foot. Warning periods (1–3.5 seconds) and inter-trial periods (6–10 seconds) varied. All participants performed 16 trials. In 25% of trials a SAS was given at the instant of the ‘go’ signal.

### Data collection

#### EMG

EMG data were collected from the tibialis anterior and rectus femoris muscles on both sides of the body, and the left sternocleidomastoid (SCM) muscle. Self-adhesive Ag-AgCl electrodes (Tyco Arbo ECG) were placed approximately 2 cm apart and longitudinally on the belly of each muscle, according to Seniam guidelines [23]. EMG signals were sampled at 2000 Hz, and full-wave rectified and low-pass filtered at 30 Hz (zero-lag, second order Butterworth filter).

#### Motion analysis

To evaluate the postural responses, reflective markers were placed using a full-body model [24]. Marker positions were recorded by an 8-camera 3D motion analysis system (Vicon Motion Systems, United Kingdom) at a sample rate of 100 Hz and low-pass filtered at 10 Hz (zero-lag, second order Butterworth filter). During the simple reaction time task, a triaxial accelerometer was placed on the foot that performed the ankle dorsiflexion movement. Accelerometer signals were sampled at 2000 Hz.

### Data analysis

#### Postural responses

For each participant, the ensemble average EMG activity during trials was calculated for each muscle, separately for trials with and without a SAS. Onset latencies of tibialis anterior and rectus femoris activity (the prime movers for the evoked postural response) were determined using the semi-automatic computer algorithm that selected the first instant at which the EMG activity exceeded a threshold of 2 standard deviations above the mean background activity, as calculated over a 500 ms period just prior to platform movement. Latencies were first selected by the computer algorithm, then visually approved or (when necessary) corrected [14]. Mean response amplitude of the ensemble average was calculated over 100 ms following the onset of muscle activity and corrected for background EMG activity. The mean onset and amplitude of tibialis anterior and rectus femoris activity in the left and right leg was taken, as there was no systematic difference between the legs; either when comparing the left and right leg, or when comparing the most and least affected leg.

Step onset and step length were determined using the position data of the heel and toe markers. Step onset was defined as the time between the start of the platform displacement and the time at which the heel and toe markers moved backwards with respect to the platform (velocity > 0,1 m/s). Step length was defined as the backward displacement of the toe markers during the step. We determined the number of balance correcting steps by visual inspection of video data.

To determine the ‘quality’ of the first balance correcting step, we calculated the angle of the stepping leg at the end of the first step (i.e. foot contact of the stepping leg)[25]. The leg angle is the angle of the line connecting the toe marker and the midpoint of the pelvis markers with respect to the vertical. A negative leg angle during backward stepping represents a situation in which the pelvis is located posterior to the stepping foot. Thus, following backward perturbations a more negative leg angle represents a more inefficient first step.

#### Startle reflex

For each trial in which a SAS was applied, we determined whether a startle reflex occurred. A startle reflex was defined as a short latency response in the SCM-muscle, starting within 130 ms following the SAS. The response had to exceed, for at least 20 ms, a threshold of 2 SD above mean background activity, as calculated over a 500 ms period just prior to the SAS.*Simple reaction time task*. Two reaction time parameters were assessed, accelerometer reaction time and EMG reaction time in tibialis anterior muscle. Onset latencies of EMG activity and foot accelerations were determined using a semi-automatic computer algorithm described above.

### Statistical analysis

Data from PD patients were analyzed using a repeated measures ANOVA, with SAS (*SAS –no SAS*) as within subjects factor and HY-stage (*HY<3—HY3*) and freezing (*freezing—non-freezing*) as between- subjects factors. In case of a significant *SASxHY-stage* or *SASxfreezing* interaction, post-hoc Student’s t-tests were performed to identify differences between subgroups.

To determine whether outcomes differed between patients and control subjects, independent of clinically-identified postural instability or freezing of gait, we compared the controls with the least affected patients (either HY<3 or non-freezers). To this aim, we performed a repeated measures ANOVA, with SAS as within subjects factor and group (*controls—least affected patients*) as between subjects factor.

Finally, in PD patients, we determined Pearson’s correlation coefficients for non-startle trials between the amplitude of tibialis anterior activity during the postural responses and (i) the step length and (ii) the leg angle. The alpha level was set at 0.05.

## Results

### Clinical assessment

Clinical characteristics of the study participants are shown in Table 1. Patients with postural instability were on average six years older than those without postural instability (t(23) = -2.186, p = 0.039); age did not differ between freezers and non-freezers (t(23) = 0.173, p = 0.864). The MDS-UPDRS-III score did not differ significantly between patients with and without postural instability (t(23) = -1.003, p = 0.326), nor between freezers and non-freezers (t(23) = -0.615, p = 0.544). In addition, the FAB-score did not differ between the subgroups (t(23)<0.768, p>0.450). Freezers had higher scores on the N-FOGQ compared to non-freezers (t(23) = -11.296, p<0.001); the N-FOGQ score did not differ between patients with and without postural instability (t(23) = -0.635, p = 0.532).

**Table 1:** Participant characteristics.

	Age (years)	Sex	UPDRS-III	No. of freezers	N-FOGQ	FAB	Disease duration (years)
HY<3	64 (55–76)	12 M, 2 F	35 (14–50)	5	7 (0–22)	15 (9–18)	10 (4–23)
HY3	70 (59–81)	8 M, 3 F	38 (23–50)	6	8 (0–22)	14 (8–18)	10 (2–16)
controls	67 (57–77)	11 M, 4 F					

*Data are mean (range)*. *UPDRS = MDS-Unified Parkinson’s disease rating scale part III (score/132)*, *N-FOGQ = New Freezing of Gait Questionnaire(score/33)*, *FAB = Frontal Assessment Battery (score/18)*.

#### Automatic postural response

A backward perturbation always resulted in a bilateral response in the tibialis anterior and rectus femoris muscles. The SAS accelerated the onset of the tibialis anterior responses in PD patients by on average 14 ms (*SAS*; F_1,21_ = 13.633, p = 0.001; Figs. 1 and 2). Latencies and their acceleration by the SAS did not differ between patients with and without postural instability (*SASxHY-stage*; F_1,21_ = 0.173; p = 0.681). However, the acceleration of tibialis anterior responses was significantly attenuated in the freezers (5 ms acceleration) compared to the non-freezers (20 ms acceleration; *SASxfreezing*; F_1,21_ = 5.150, p = 0.034; Fig. 2). Post-hoc analysis revealed that latencies during trials without a SAS did not differ between freezers and non-freezers (t(23) = -0.391, p = 0.699), whereas with a SAS, they were significantly delayed in the freezers compared to non-freezers (t(23) = -2.447, p = 0.022). Non-freezers did not differ from controls (*Group*; F_1,27_ = 0.107; p = 0.746; *SASxGroup*; F_1,27_ = 0.210, p = 0.651). The same pattern was seen for the rectus femoris muscle. The SAS accelerated the onset of the postural responses in PD patients by on average 10 ms (*SAS*; F_1,21_ = 10.743, p = 0.004). The acceleration did not differ significantly between patients with and without postural instability (*SASxHY-stage*; F_1,21_ = 1.247; p = 0.277), but was significantly reduced in the freezers (2 ms acceleration) compared to the non-freezers (14 ms acceleration; *SASxFreezing*; F_1,21_ = 6.473, p = 0.019). Post-hoc analysis revealed that latencies during trials without a SAS did not differ between freezers and non-freezers (t(23) = -1.439, p = 0.164), whereas they were significantly delayed in the freezers compared to non-freezers following SAS presentation (t(23) = -2.416, p = 0.043). Non-freezers did not differ from controls (158±13, 18 ms acceleration, *Group*; F_1,27_ = 0.013; p = 0.909; *SASxGroup*; F_1,27_ = 0.544, p = 0.467).

**Fig 1:** Average EMG-activity recorded in the tibialis anterior muscle of a single PD-patient (with freezing of gait and postural instability) during backward balance perturbations. Grey line represents perturbations with SAS (determined onset latency = 140 ms). Black line represents perturbations without SAS (determined onset latency = 145 ms).

**Fig 2:** Mean onset latencies (SE) of the automatic postural response in tibialis anterior (TA). HY = Hoehn and Yahr stage. A SAS significantly accelerated automatic postural responses. Latencies and their acceleration by the SAS did not differ between patients with and without postural instability. The SAS-induced acceleration of tibialis anterior responses was significantly attenuated in the freezers compared to the non-freezers. Non-freezers did not differ from controls.

The SAS had no effect on the amplitudes of tibialis anterior or rectus femoris activity (*SAS*; F_1,21_ = 1.105, p = 0.305; *SAS*; F_1,21_ = 2.122, p = 0.160, respectively). Tibialis anterior amplitudes were on average 40% smaller in patients with postural instability compared to patients without postural instability (*HY-stage*; F_1,21_ = 7.308, p = 0.013; Fig. 3), whereas they did not significantly differ between freezers and non-freezers (*Freezing;* F_1,21_ = 2.963, p = 0.100). Rectus femoris amplitudes were on average 21% smaller in patients with postural instability compared to patients without postural instability, but this difference did not reach significance due to large within- and between-subjects variability (*HY-stage*; F_1,21_ = 0.588, p = 0.452). Rectus femoris amplitudes did not differ between freezers and non-freezers either (*Freezing*; F_1,21_ = 0.159, p = 0.694). In addition, amplitudes of tibialis anterior and rectus femoris responses did not differ between patients without postural instability and controls (*Group*; F_1,27_ = 0.122; p = 0.729; *Group*; F_1,27_ = 1.634; p = 0.212, respectively).

**Fig 3:** Mean amplitudes (SE) of the automatic postural response in tibialis anterior (TA). HY = Hoehn and Yahr stage. Tibialis anterior amplitudes were significantly smaller in patients with postural instability compared to patients without postural instability, whereas they did not significantly differ between freezers and non-freezers. Amplitudes of tibialis anterior did not differ between patients without postural instability and controls.

#### Balance correcting step

Step onset did not differ between patients with and without postural instability (*HY-stage*; F_1,21_ = 0.001, p = 0.971; Table 2), nor between freezers and non-freezers (*Freezing*; F_1,21_ = 0.079, p = 0.782). The SAS had no general effect on the step onset (*SAS*; F_1,21_ = 0.988, p = 0.332). In the freezers, however, we observed later step onsets in trials with a SAS, whereas non-freezers demonstrated an earlier step onset, yielding a significant *SASxFreezing* interaction (F_1,21_ = 6.614, p = 0.018). Step onset did not differ between non-freezers and controls (*Group;* F_1,27_ = 0.007, p = 0.936).

Patients with postural instability had smaller step lengths (12±5 cm) than patients without postural instability (20±7 cm; *HY-stage*; F_1,21_ = 6.815, p = 0.016; Fig. 4), but step length did not differ between freezers and non-freezers (*Freezing*; F_1,21_ = 2.810, p = 0.109; Table 2). A SAS did not influence step length (*SAS*; F_1,21_ = 2.537, p = 0.126). Step lengths were shorter in patients without postural instability compared to controls (26±4 cm; *Group;* F_1,27_ = 8.261; p = 0.008; Fig. 4). The quality of the balance correcting step was lower in patients with postural instability compared to patients without postural instability as evidenced by more negative leg angles (-10.7±5.0^0^ vs -4.6±3.9^0^; *HY-stage*; F_1,21_ = 7.060; p = 0.015; Fig. 4). Leg angles did not differ between freezers and non-freezers (*Freezing*; F_1,21_ = 1.602, p = 0.219). The SAS improved the leg angle in PD patients by on average 0.9^0^ (*SAS*; F_1,21_ = 10.121, p = 0.004; Fig. 4) with no differences between patients with and without postural instability (*SASxHY-stage*; F_1,21_ = 1.757, p = 0.199) or between patients with and without freezing of gait (*SASxFreezing*; F_1,21_ = 0.102, p = 0.753). Patients without postural instability had more negative leg angles compared to controls (*Group*; F_1,27_ = 11.884, p = 0.002; Fig. 4). Patients with postural instability needed more steps to recover from the balance perturbations than patients without postural instability (*HY-stage*; F_1,21_ = 4.765, p = 0.041; see Table 2). The average number of balance correcting steps tended to be higher in freezers compared non-freezers, but differences were not significant (*Freezing*; F_1,21_ = 3.920, p = 0.061). The SAS did not influence the number of steps (*SAS*; F_1,21_ = 0.830, p = 0.373). Patients without postural instability made more steps compared to control subjects (*Group*; F_1,27_ = 4.343, p = 0.047).

In PD patients, the leg angle correlated strongly with step length (r_p_ = 0.887; p<0.001) and moderately with response amplitudes in tibialis anterior (r_p_ = 0.444; p = 0.026). Correlations between step length and tibialis anterior amplitudes bordered significance (r_p_ = 0.377; p = 0.063).

**Fig 4:** Mean step lengths and leg angles (SE) during backward perturbations. Patients with postural instability had significantly smaller step lengths than patients without postural instability, but step length did not differ between freezers and non-freezers. Step lengths were significantly shorter in patients without postural instability compared to controls. Leg angles were significantly smaller in patients with postural instability compared to patients without postural instability. Leg angles did not differ between freezers and non-freezers. Patients without postural instability had more negative leg angles compared to controls.

**Table 2:** Step onset and number of balance correcting steps.

	Step onset (ms)		Number of steps	
	No SAS	SAS	No SAS	SAS
Controls	349±51	337±45	1.3±0.4	1.3±0.4
HY<3	347±53	340±57	1.6±0.6	1.8±0.7
HY3	351±45	345±58	2.5±0.8	2.3±0.6
freezers	337±57	363±51	2.4±0.8	2.3±0.7
non-freezers	346±58	337±46	1.7±0.7	1.8±0.6

*Values are mean (SD)*.

### Correlation between StartReact effects and underscaling

In PD patients, SAS-induced acceleration of postural responses in the tibialis anterior muscle did not correlate with the amplitude of tibialis anterior activity (r_p_ = 0.026; p = 0.902), nor with step length (r_p_ = -0.078; p = 0.711) or leg angle (r_p_ = -0.052; p<0.806).

### Association between startle reflexes and StartReact

Following balance perturbations with a SAS, we found no difference in startle reflex occurrence between freezers (23% of trials with SAS), non-freezers (38%), and controls (23%; F_2,39_ = 0.504, p = 0.608). Furthermore, more frequent occurrence of startle reflexes was not associated with a larger StartReact effect in individual participants, neither in tibialis anterior (r_p_ = 0.194, p = 0.230) nor in rectus femoris (r_p_ = 0.045, p = 0.784). To further investigate the relation between the presence of SCM-reflexes and onset latencies in the TA-muscles during SAS-trials, we determined the onset of TA-responses for each SAS-trial separately. We conducted an ANOVA to compare SAS-induced accelerations in TA onsets between trials with and without SCM reflex. We included g*roup (freezers—non-freezers—controls*) as a between-subjects factor. As participants could either have SCM+ trials only, SCM- trials only or a combination of both, we also included the presence of *SCM reflex (yes/no)* as a between-subjects factor. This analysis demonstrated that overall, accelerations in TA onset latencies did not differ between trials with and without SCM activation (13±4 ms vs. 16±4 ms; *SCM reflex*, F_1,49_ = 0.321, p = 0.573); g*roup x SCM reflex*, F_2,49_ = 0.280, p = 0.757; see Fig. 5). Post-hoc LSD tests confirmed the reduced SAS-induced acceleration in the freezers compared to the non-freezers (p = 0.043), as well as the absence of differences between non-freezers and controls (p = 0.794).

**Fig 5:** Mean acceleration (SE) of onset latencies of automatic postural responses in tibialis anterior (TA) during SAS-trials with and without a startle reflex in the sternocleidomastoid (SCM) muscle. The number of participants who showed trials with and without SCM reflexes is indicated on top of each bar. In all groups, acceleration of responses did not differ significantly between SAS-trials with and without a startle reflex in the SCM-muscle.

### Simple reaction time task

In the ankle dorsiflexion task, the StartReact effect was significantly attenuated in the freezers compared to the non-freezers, which was reflected both in the latencies of tibialis anterior activity (20 ms acceleration for freezers, 45 ms for non-freezers; *SASxFreezing*; F_1,21_ = 25.651, p<0.001, see Table 3) and in the accelerometer onset (18 ms acceleration for freezers, 50 ms for non-freezers; *SASxFreezing*; F_1,21_ = 13.413, p<0.001). There were no differences in acceleration between patients with and without postural instability, neither in the EMG responses (*SASxHY-stage*; F_1,21_ = 0.133, p = 0.719) nor in the accelerometer onset (*SASxHY-stage*; F_1,21_<0.001, p = 0.999).

**Table 3:** Ankle dorsiflexion.

	Onset TA (ms)		Onset accelerometer (ms)	
	No SAS	SAS	No SAS	SAS
Control subjects	140±16	98±18	156±22	109±16
HY<3	135±15	98±18	151±24	112±25
HY3	138±13	108±12	155±20	123±11
freezers	131±11	111±12	144±17	126±15
non-freezers	141±14	96±16	160±24	110±22

*Values are mean (SD)*. *HY = Hoehn and Yahr stage*.

## Discussion

We examined postural responses with and without a startling acoustic stimulus (SAS) in a carefully selected group of PD patients, and specifically contrasted the results between patients with pronounced postural instability versus those without, and between those with FOG versus those without, while statistically controlling for the potential confounding effects of the other factor. Using this method, we were able to delineate characteristics specific to postural instability, and factors specific to freezing of gait. The results of the present study reveal a distinct dissociation between postural instability and FOG. We found reduced amplitudes of automatic postural responses following a backward perturbation, as well as reduced length and quality of the first balance correcting step, in patients with postural instability compared to patients without postural instability. These parameters did not differ between freezers and non-freezers. In contrast, the accelerating effect of a SAS on both postural responses and simple ankle dorsiflexion movements was not different between patients with and without postural instability. Instead, this effect was selectively attenuated in the freezers, whereas it was completely intact in non-freezers. The dissociation between postural instability and FOG was also evident from the lack of associations between StartReact effects and underscaling of balance correcting responses.

### Different mechanisms underlie freezing and postural instability

The frequent co-existence of freezing of gait and postural instability has raised the possibility of a shared pathophysiology [1, 2, 4, 26]. Indeed, this view is supported by previous studies that reported profound underscaling of balance correcting responses in freezers [27], as well as a defective StartReact effect [3, 5]. The present findings, however, strongly argue against the suggestion of a common underlying mechanism. The assessment of balance correcting responses combined with a StartReact paradigm in a carefully balanced group of PD patients enabled us to identify hypometric balance correcting responses being specific to postural instability, versus defective StartReact being specific to freezing. The absence of correlations between SAS-induced accelerations of postural responses and continuous markers of postural instability such as amplitudes of postural responses, step length and leg angles particularly speaks in favor of dissociated mechanisms.

### Underscaling of balance responses underlies postural instability

Patients with evident postural instability (HY3) had smaller amplitudes of automatic postural responses and a reduced length of the balance correcting step compared to patients without evident postural instability (HY<3). This resulted in a lower quality of the first balance correcting step, as reflected by more negative leg angles and larger numbers of steps needed to recover from the balance perturbations. These findings are in line with previous studies that also reported similar underscaling of balance correcting responses (including stepping) in PD patients compared to controls [27–31]. These studies, however, did not differentiate between H&Y stages. Importantly, the present results show that not only patients with evident postural instability, but also those without (clinically-defined) postural instability had smaller balance correcting steps and poorer step quality compared to healthy controls. The significant correlations of hypometric response amplitudes and step lengths with step quality highlight the degree of underscaling being the critical determinant of PD-related balance impairments.

The observation of underscaled balance correcting responses in PD patients without evident postural instability is indicative of a continuum of balance impairments in PD, which calls for more sensitive clinical tests to identify and monitor these impairments.

The precise mechanisms underlying the underscaling of balance correcting responses are not completely clear. Moreover, it is unknown whether the underlying mechanisms are the same for hypometric postural responses and for reduced step lengths. The observation that step length tended to correlate with postural response amplitude may point at a common pathophysiological mechanism. Although automatic postural responses and stepping responses are organized in different neural structures, the cortex and basal ganglia are involved in shaping both to the demands of the task at hand [32]. The underscaling may thus reflect the hypokinesia that characterizes PD [33], which presumably results from abnormal proprioceptive-motor integration in the supplementary motor cortex [28, 34]. This explanation, however, raises the question why dopaminergic medication has only a small [30, 35] or no effect [29, 36, 37] on balance responses, whereas it is able to improve supplementary motor cortex activity [38]. The minor effects of dopaminergic medication on balance impairments could indicate that lesions in non-dopaminergic pathways primarily underlie postural instability in PD. Deficiencies in cholinergic pathways might be considered, as degeneration of cholinergic neurons is associated with falls [2], and treatment with the acetylcholinesterase inhibitor donepezil reduced the number of falls in PD patients [39]. Moreover, bilateral lesioning of the cholinergic part of the PPN in monkeys induced postural deficits [2]. In humans, postural instability in PD is correlated with both electrophysiological [40] and PET-imaging [41, 42] measures of PPN-cholinergic dysfunction. Although deficits in non-dopaminergic pathways seem to be of great importance with regard to balance impairments in PD, the marginal effects of dopaminergic medication do not necessarily preclude a role for dopamine deficiency in the underlying pathophysiology, because the threshold for therapeutic relief may simply be higher than for other symptoms [43]. Hence, future studies should further investigate the role of dopaminergic as well as non-dopaminergic pathways in the underscaling of balance correcting responses.

### Disturbed StartReact in freezers

In both PD patients and controls, a smaller SAS-induced acceleration was observed during postural responses compared to the ankle dorsiflexion task, which is in line with the literature [14, 44, 45]. There is, however, strong evidence that postural responses to balance perturbations are preprogrammed and subject to triggered release by a SAS, resulting in a StartReact effect [14, 46, 47]. The smaller degree of acceleration by a SAS might be explained by differences in neural organization. In contrast to voluntary reactions in response to an imperative auditory or visual stimulus, automatic postural responses do not involve transcortical pathways [32, 48, 49], but are likely encoded by assemblies of neurons in the pmRF [6]. The observation of defective StartReact effects in freezers is novel for automatic postural responses following backward balance perturbations. Previous studies demonstrated similar results for simple ballistic movements of the upper and lower extremities and when initiating gait [3, 5]. The consistency of these findings in different tasks suggests a common origin, possibly involving dysfunction of upper brainstem structures [2, 3]. Here, we extend on these findings by showing that defective StartReact is specific to freezing of gait and is not related to postural instability.

The occurrence of the StartReact effect critically depends on the upcoming movement being readily prepared and ‘stored’. The exact neural structures involved remain to be unraveled [8], but there is accumulating evidence that StartReact reflects direct release of subcortically stored motor programs, possibly from the pontomedullary reticular formation (pmRF)[7, 10]. Our group investigated the StartReact effect in patients with hereditary spastic paraplegia (HSP). Patient with HSP have retrograde axonal degeneration of the corticospinal tract [50, 51], while the reticulospinal tract is not affected [44]. In these patients, ankle dorsiflexion reaction times to a visual stimulus were delayed, which finding concurred with delayed corticospinal motor conduction times as measured with supramaximal TMS. Upon the presentation of a visual stimulus combined with a SAS, however, they exhibited similar latencies to healthy control subjects, irrespective of the presence of a SCM-reflex.

Based on this notion of a SAS-induced release of subcortical motor program, the defective StartReact effect in freezers may either indicate poor movement preparation at this levelor reduced responsiveness of these structures to triggers releasing the prepared motor responses. Finally, the attenuated StartReact effect in patients with FOG can be the result of an increased gain of the reticulospinal output [11]. In freezers, the gain of the reticulospinal output might be set at maximum to compensate for underlying degenerative changes. In that case, the gain cannot increase further and the SAS will have no additional effect on a voluntary reaction time task, such as the present ankle dorsiflexion task, nor on corrective postural responses. However, our results on the effects of a SAS on the scaling of responses do not seem to argue in favor of differences in gain underlying the attenuated StartReact effects in freezers. Stepping leg angles significantly improved when the SAS was applied together with the perturbation, which effect was similar between freezers and non-freezers. Furthermore, in our previous paper on StartReact effects in gait initiation, we reported greater amplitudes for anticipatory postural adjustments as well as greater response amplitudes in the tibialis anterior in trials with a SAS compared to those without [52]. Again, these effects of the SAS on response scaling were not different between freezers and non-freezers, whereas the effects of the SAS on response onsets were similar to those presently reported.

Importantly, there are several observations that suggest that startle reflexes and StartReact effects are at least partly dissociated. First, while a prepulse at 100 ms and 500 ms was shown to significantly reduce the amount of SCM activation, the StartReact effect was reported to be unaffected by the prepulse [53]. Second, the presence of a startle reflex in SCM does not appear to be a prerequisite for the StartReact effect. Although some studies [54–56] reported an attenuation of StartReact effects when no startle reflex activity is observed, several other studies could not establish a significant relationship between the occurrence of SCM responses and StartReact, which was true both for experiments involving simple reaction time tasks [7, 57] and for tasks involving gait and postural responses [7, 14, 58–61]. As a SAS restored reaction times in patients with HSP, irrespective of the presence of a SCM-reflex, startle reflexes are likely not a prerequisite for a SAS-induced release of a subcortically stored motor programs. A final observation in support of (at least partly) dissociated mechanism underlying startle reflexes and StartReact comes from a study that reported on the effect of PPN-stimulation in PD patients with FOG [3]. When the stimulator was turned off, the StartReact effect and startle reflexes were absent in these patients, but PPN-stimulation restored StartReact effects, while leaving the impairment in startle reflexes unchanged. This implies that a defective StartReact effect in freezers does not merely represent a degradation of primary startle reflex pathways, but rather points at a specific motor preparation deficit.

Remarkably, the putative inadequate representation or release of motor programs at brainstem level in freezers did not result in delayed postural responses, despite the fact that these responses are presumably mediated also by neurons in the pmRF [6, 10]. Given the great complexity of neuronal organization at the brainstem level, and uncertainties regarding the integrative role of brainstem nuclei in the generation of movement, we can only speculate about a possible explanation for this rather unexpected result. Possibly, the postural response is released from different (brainstem) neurons when triggered by a SAS as compared to the proprioceptive input induced by the mechanical perturbation itself. This implies that some neurons may be primarily involved in the preparation of the automatic postural response, whereas others are responsible for its release by afferent information. By analogy with voluntary movements, the SAS could have access to neurons that are involved in the preparation of the response [10]. In freezers, these preparatory structures may be defective, whereas the neural circuits involved in the release of automatic postural responses by proprioceptive input may be intact. Further research should identify the existence of such brainstem networks in order to support this hypothesis.

In conclusion, our results suggest that the mechanisms underlying freezing of gait and postural instability in PD patients are at least partly different. This stresses the notion that future studies should address gait and balance separately [62], and calls for studies elucidating the specific neural circuits subserving these behaviors, as well as their degradation in PD. Novel paradigms, such as motor imagery of balance control and gait [63], could help to further unravel the separate mechanisms underlying postural instability and FOG.
